# Correlation of Dynamic PET and Gene Array Data in Patients with Gastrointestinal Stromal Tumors

**DOI:** 10.1100/2012/721313

**Published:** 2012-06-04

**Authors:** Ludwig G. Strauss, Antonia Dimitrakopoulou-Strauss, Dirk Koczan, Leyun Pan, Peter Hohenberger

**Affiliations:** ^1^Medical PET Group, Biological Imaging, CCU Nuclear Medicine, German Cancer Research Center, 69120 Heidelberg, Germany; ^2^Molecular Immunology Group, Institute of Immunology, University of Rostock, 18055 Rostock, Germany; ^3^Division of Surgical Oncology and Thoracic Surgery, Department of Surgery, Mannheim University Medical Center, University of Heidelberg, 69135 Mannheim, Germany

## Abstract

*Introduction*. The results obtained with dynamic PET (dPET) were compared to gene expression data obtained in patients with gastrointestinal stromal tumors (GIST). The primary aim was to assess the association of the dPET results and gene expression data. *Material and Methods*. dPET was performed following the injection of F-18-fluorodeoxyglucose (FDG) in 22 patients with GIST. All patients were examined prior to surgery for staging purpose. Compartment and noncompartment models were used for the quantitative evaluation of the dPET examinations. Gene array data were based on tumor specimen obtained by surgery after the PET examinations. *Results*. The data analysis revealed significant correlations for the dPET parameters and the expression of zinc finger genes (znf43, znf85, znf91, znf189). Furthermore, the transport of FDG (k1) was associated with VEGF-A. The cell cycle gene cyclin-dependent kinase inhibitor 1C was correlated with the maximum tracer uptake (SUVmax) in the tumors. *Conclusions*. The data demonstrate a dependency of the tracer kinetics on genes associated with prognosis in GIST. Furthermore, angiogenesis and cell proliferation have an impact on the tracer uptake.

## 1. Introduction

 Gastrointestinal stromal tumors (GIST) are rate tumors arising in the gastrointestinal tract. Imatinib mesylate (imatinib) is frequently used in these patients for treatment. However, the resection of the tumor is the primary aim of treatment. Frequently, mutations are noted in the kit or platelet-derived growth factor receptor-A (PDGFRA). The expression of genes and their possible mutations are important for treatment of GIST. The survival is primarily correlated with the stage of disease, the tumor size, and the proliferation. Rutkowski et al. differentiated the GIST according to location and stage and reported about a 5-year survival rate in gastric GIST of 96% for stage IA, 92% for IB, 51% for II, 22% for IIIA, and 22% for IIIB [1]. Setoguchi et al. evaluated the prognostic aspect of gene array data in GIST [2]. The authors were able to show that VCAN and CD9 are prognostic markers in gastric GIST. Disease-free survival was significantly longer for patients if CD9 was enhanced and expressed, and VCAN revealed a low expression. Another study by Schmieder et al. demonstrated that p16 is also important for the identification of high-risk GIST and p16 was predictive for poor outcome [3]. The literature results demonstrate that quantitative data about the expression of genes may be helpful to gain prognostic information.

 Positron emission tomography (PET), in particular PET-CT, can be used to obtain accurate information about the distribution of a tracer over time within a given volume if a dynamic acquisition, for example, for one hour is performed. Dynamic PET (dPET) and PET-CT (dPET-CT) data can be analyzed by applying compartment and non-compartment models to achieve detailed information about the tracer kinetics.

 F-18-deoxyglucose (FDG) is the most commonly used tracer for PET in oncology. The tracer kinetics of FDG is closely dependent on the expression of glucose transporters and hexokinases. However, it was shown that the kinetics of FDG may be modulated by genes associated with angiogenesis and proliferation [4, 5]. Thus, gene expression may be predicted from a detailed analysis of the FDG kinetics in certain tumors. However, no data exist about the correlation of gene expression and quantitative dynamic PET data in GIST. Therefore, the aim of this study was to assess the association of FDG kinetics and gene expression in GIST.

## 2. Material and Methods

 The study comprises 22 patients with GIST scheduled for surgery. Dynamic PET studies were performed prior to surgery within the routine diagnostics for tumor staging. All patients had pretreatment with imatinib, and surgery was intended to remove the tumor tissue. The body volume for the dynamic study had been determined according to the clinical information where the surgery was performed. Following the intravenous injection of 200–300 MBq FDG, a dynamic data acquisition was initiated for one hour. Then whole body imaging was performed following the dynamic study. The dynamic study comprises 28 frames, including 10 frames of 30 s, 5 frames of 60 s, 5 frames of 120 s, and 8 frames of 300 s. Following the iterative image reconstruction, the images were converted to standardized uptake value (SUV) images for further evaluation. The SUV was calculated according to the following: SUV = tissue concentration (Bq/g)/(injected dose (Bq)/body weight (g) [6].

 In 20 of the 22 patients the dynamic studies could be evaluated using a 2-tissue-compartment model. Volumes of interest (VOI) were used for the quantitative assessment of the tumors. The quantitative evaluation was performed with a dedicated software and included the calculation of SUV and the maximum SUV. Furthermore, the tracer kinetics was analyzed using a 2-tissue-compartment model. For this purpose a VOI was placed over the descending aorta to obtain an input function for the model. It was already shown by Ohtake et al. that the input data for FDG can be obtained via VOIs from a large vessel with high accuracy [7]. The authors noted a median error of 3.75% for the image-derived results as compared to the arterial sampling data. No partial volume correction was needed, because the diameters of the vessels exceeded 8 mm, which correlates with a recovery factor of 0.85 for our system and the image reconstruction settings used for the study. The compartment analysis software provides five parameters: *k1* and *k2*, associated with the transport of FDG; *k3* and *k4*, which are associated with the phosphorylation and dephosphorylation; vb, the fractional blood volume of a VOI, also referred to as vessel density. Furthermore, a noncompartment model was applied to the data to obtain the fractal dimension (FD) of the time activity data. The positioning of the VOIs was done according to the information provided by the surgeons about the location, where the tissue specimen was removed from the tumor. Thus, we tried to get the quantitative dPET data spatially close to the region where the tissue specimen was obtained.

 Tumor resection was performed in the 22 patients. A small fraction of the tumor was used for gene array analysis. The tissue specimens were immediately stored in liquid nitrogen, and total RNA was extracted for further processing. The quality of isolated RNA was evaluated photometrically using the 280/260 ratio and on an agarose gel. We used the U133A 2.0 gene array (Affymetrix Inc., Santa Clara, CA, USA), which provides quantitative information about 54675 gene probes. The processing of the RNA and gene arrays was done according to the manufacturer's recommendations. Gene chip expression data were normalized for the beta-2 microglobulin (Affymetrix code 34644_at, Homo sapiens mRNA for beta-2 microglobulin) using the following equation: relative expression value (REV) = 1,000 × expression value of a gene/expression value for beta-2 microglobulin [8].

 The statistical evaluation was performed with Stata/SE 11.2 (Stata Corporation, College Station, TX, USA) on a Mac Pro 2 × 2.93 GHz, 12 Core Intel Xeon system with 24 GB RAM using Mac OS X 10.7.3 (Apple, Cupertino, CA, USA). The same system was also used for all data processing tasks, including dPET and gene array data. A dedicated software (GenPET), developed by our group, was used for the correlative evaluation of dynamic PET and gene array data [9]. The software provides the correlative assessment of both PET and gene array data. For the correlation analysis, a significance level of *P* < 0.05 was used. Based on the significant results of the correlation analysis, nonlinear regression functions were calculated for the gene array and PET data.

## 3. Results

 The statistical data for the PET parameters are provided in Table 1. The mean SUV was 6.597, nearly half of the SUV_max_. The fractional blood volume (vb), associated with the vessel density, was 0.108, which reflects about 11% of the tumor volume evaluated by VOIs. The maximum vb was 0.253, which refers to a blood volume fraction of about 1/4 of the tumor volume. As expected, *k1* (FDG transport) was high, and *k3* (FDG phosphorylation) was relatively low in these tumors.

 Several studies are focused on the gene expression patterns in GIST. Rink et al. compared the gene expression signatures with the response to imatinib mesylate treatment in 63 patients [10]. Overall, the authors report about 38 genes, which were expressed lower prior to therapy and were associated with response to treatment. Interestingly, 18 of the 38 genes are related to the genes of the zinc finger group. The function of all zinc finger genes is not well known, but it is likely that they are involved in signaling and cell regulation mechanisms. Based on the results from Rink et al., we evaluated the zinc finger gene data for possible correlations with the PET data. We used a nonlinear regression approach and combinations of two or three PET variables for the correlation/regression analysis. Significant correlations (*r* > 0.8) were found for znf43, znf85, znf91, and znf189. The PET variables used for the nonlinear regression functions are shown on the *x*-axis in Figure 1, while the *y*-axis reflects the corresponding gene expression data (unit for gene expression data: REV).

Besides the zinc finger genes, we noted also a significant difference for high (>0.441) and low *k1* values and the expression of VEGF-A, an angiogenesis-related gene (Figure 2). Interestingly, this had been already reported, for example, for colorectal tumors and gene array data [4]. The cyclin-dependent kinase inhibitor 1C has an impact on cell proliferation and acts as a tumor suppressor gene. A correlation (*r* = 0.85) was noted for this gene and the maximum SUV (Figure 3).

## 4. Discussion

 In patients with GIST, PET with FDG is a common procedure for both, diagnostic purpose for staging and follow to assess the response to treatment. Apostolopoulos et al. evaluated 65 dynamic PET-FDG studies in patients with liver metastases from GIST [11]. He used parametric imaging for the data evaluation and report about an accuracy of 87.7% and a sensitivity of 88.2%. Gayed et al. examined 54 patients with PET-FDG and reported about a sensitivity of 86% [12]. The results demonstrate that PET is useful to identify GIST lesions.

 Dynamic PET studies provide the assessment of details of the tracer kinetics using compartment and noncompartment models. The 2-tissue-compartment model is the standard for the assessment of FDG dynamic data. One major advantage of dPET is the possibility to obtain the input function for the 2-tissue model from the images without arterial blood sampling. We calculated all five parameters of the model using a dedicated software developed by our group. The software uses a modified support vector machines algorithm to calculate the model parameters. The dephosphorylation rate of FDG may be low in tumors, but we included *k4* also in the model calculations to achieve most accurate results.

 One aspect of major importance is the correlation of PET results with molecular biological data. Park et al. compared in 26 patients with gastric GIST the maximum SUV (SUV_max_) with the Ki-67 index [13]. The authors obtained a correlation of *r* = 0.854 for the two parameters. Based on our results, the SUV_max_ was generally enhanced and above 10 SUV. The compartment data suggested a primary contribution of vb and *k1* to the global FDG uptake. However, more data are needed to evaluate the dependency of the global uptake and maximum uptake on tumor proliferation.

 Rink et al. identified genes, correlated with response to imatinib mesylate treatment [10]. Most of the genes were zinc finger genes. These genes are usually associated with the regulation of transcription. We noted significant correlations for the PET parameters and ZNF43, ZNF85, ZNF91, and ZNF189 (Figure 1). Primarily, the SUV and SUV_max_ were correlated with the zinc finger genes. However, SUV and SUV_max_ alone correlate only with ZNF189; therefore, the results from the dPET are required to predict the gene expression accurately. Rink et al. were able to demonstrate that a subgroup of zinc finger genes are predictive for the treatment outcome in patients treated with imatinib mesylate [10]. Furthermore, they performed knock down experiments, for example, with ZNF43, ZNF85, and ZNF91, and they showed that depletion of each of the ZNFs resulted in an improved sensitization to imatinib mesylate. Thus, predicting the expression of these genes from quantitative, dynamic PET results may be a promising approach for an improved evaluation of treatment response in GIST.

 Besides the zinc finger genes, other genes, for example, associated with angiogenesis, are important for the treatment results. We noted a significant difference for high and low *k1* data and the expression of VEGF-A (Figure 2). The difference of the two groups is significant with *P* < 0.0197. The same limit for *k1* (0.441) was used as in the publication about colorectal tumors and PET [4]. Therefore, it can be assumed that *k1* is generally modulated by VEGF-A expression. Overall, tumors with a *k1* less than 0.441 had a lower expression of VEGF-A as compared to tumors with a higher *k1*. However, this should be shown also for other tumor types, but we can assume that the dependency of *k1* on the VEGF-A expression is most likely not dependent on the tumor type. Thus, *k1* may be used as a general classification parameter to predict VEGF-A expression in a malignant lesion.

 The role of the cyclin-dependent kinase inhibitor 1C (cdki 1C) is described in detail in the review paper of Kavanagh and Joseph [14]. cdki 1C is involved in several regulatory processes, including tumor differentiation and angiogenesis, apoptosis, cell invasion, and metastasis. The gene acts as a tumor suppressor gene. Therefore, we noted a lower expression of cdki 1C with higher SUV_max_ values (Figure 3). Actually, no publications exist about cdki 1C and FDG in PubMed, so it is not possible to compare our results with others. Actually it can be expected that inhibitors of the cell cycle usually reveal a negative correlation to PET parameters. Based on our results in colorectal carcinoma, we were able to show that cdki 2B was negatively correlated with *k3* [5]. In contrast, cdk2 was positively correlated with the SUV in these tumors. Overall, the correlation between cdki 1C and SUV_max_ is in agreement with the conclusions of Park et al. who found a correlation for the SUV_max_ and ki-67 [10]. Thus, the SUV_max_ is likely to be predictive for tumor proliferation in GIST.

## Figures and Tables

**Figure 1:** Correlations and nonlinear regression functions of PET parameters, obtained from the dynamic studies, and gene expression data.

**Figure 2:** Low *k1* (less than 0.441) values are associated with a low expression of VEGF-A.

**Figure 3:** Correlation of the maximum SUV with cdki 1C (*r* = 0.8539).

**Table 1:** Statistical data for the PET parameters.

	SUV	SUV_max_	vb	*k1*	*k2*	*k3*	*k4*	fd	influx
Mean	6.597	13.029	0.108	0.446	0.787	0.070	0.004	1.306	0.036
Median	6.599	12.104	0.066	0.423	0.802	0.067	0.001	1.448	0.030
Minimum	1.406	2.286	0.028	0.199	0.542	0.003	0.000	1.035	0.003
Maximum	16.935	29.280	0.253	0.801	0.928	0.188	0.013	1.448	0.105
no.	20	20	20	20	20	20	20	20	20

## References

[1] Rutkowski P, Wozniak A, Debiec-Rychter M (2011). Clinical utility of the new American Joint Committee on Cancer staging system for gastrointestinal stromal tumors: current overall survival after primary tumor resection. *Cancer*.

[2] Setoguchi T, Kikuchi H, Yamamoto M (2011). Microarray analysis identifies versican and CD9 as potent prognostic markers in gastric gastrointestinal stromal tumors. *Cancer Science*.

[3] Schmieder M, Wolf S, Danner B (2008). p16 expression differentiates high-risk gastrointestinal stromal tumor and predicts poor outcome. *Neoplasia*.

[4] Strauss LG, Koczan D, Klippel S (2008). Impact of angiogenesis-related gene expression on the tracer kinetics of 18F-FDG in colorectal tumors. *Journal of Nuclear Medicine*.

[5] Strauss LG, Koczan D, Klippel S (2011). Impact of cell-proliferation-associated gene expression on 2-deoxy-2-[ ^18^F]fluoro-D-glucose (FDG) kinetics as measured by dynamic positron emission tomography (dPET) in Colorectal Tumors. *Molecular Imaging and Biology*.

[6] Strauss LG, Conti PS (1991). The applications of PET in clinical oncology. *Journal of Nuclear Medicine*.

[7] Ohtake T, Kosaka N, Watanabe T (1991). Noninvasive method to obtain input function for measuring tissue glucose utilization of thoracic and abdominal organs. *Journal of Nuclear Medicine*.

[8] Strauss LG, Dimitrakopoulou-Strauss A, Koczan D (2004). 18F-FDG kinetics and gene expression in giant cell tumors. *Journal of Nuclear Medicine*.

[9] Strauss LG, Pan L, Koczan D (2007). Fusion of positron emission tomography (PET) and gene array data: a new approach for the correlative analysis of molecular biological and clinical data. *IEEE Transactions on Medical Imaging*.

[10] Rink L, Skorobogatko Y, Kossenkov AV (2009). Gene expression signatures and response to imatinib mesylate in gastrointestinal stromal tumor. *Molecular Cancer Therapeutics*.

[11] Apostolopoulos DJ, Dimitrakopoulou-Strauss A, Hohenberger P, Roumia S, Strauss LG (2011). Parametric images via dynamic 18F-fluorodeoxyglucose positron emission tomographic data acquisition in predicting midterm outcome of liver metastases secondary to gastrointestinal stromal tumours. *European Journal of Nuclear Medicine and Molecular Imaging*.

[12] Gayed I, Vu T, Iyer R (2004). The role of ^18^F-FDG PET in staging and early prediction of response to therapy of recurrent gastrointestinal stromal tumors. *Journal of Nuclear Medicine*.

[13] Park JW, Cho CH, Jeong DS, Chae HD (2011). Role of F-fluoro-2-deoxyglucose positron emission tomography in gastric GIST: predicting malignant potential pre-operatively. *Journal of Gastric Cancer*.

[14] Kavanagh E, Joseph B (2011). The hallmarks of CDKN1C (p57, KIP2) in cancer. *Biochimica et Biophysica Acta*.

